This article has been retracted.

# Colloid Cyst: A Potentially Life-Threatening Etiology of Severe Headache in a Patient With Migraine

**DOI:** 10.7759/cureus.18424

**Published:** 2021-10-01

**Authors:** Rayan N Alshuaylan, Abdulelah A Alismail, Fisal M Haobani, Mohammed R Alfulayw, Abdullah Y Abu Maghayed, Alya A Khashoggi, Shahid A Al-Mahdi, Sarah A AlKishi, Jawad H Alnaqaa, Shahad B Alwazzan, Malak Alshammari

**Affiliations:** 1 College of Medicine, Shaqra University, Shaqra, SAU; 2 College of Medicine, King Faisal University, Al-Ahsa, SAU; 3 College of Medicine, Vision Colleges, Riyadh, SAU; 4 College of Medicine, Imam Abdulrahman Bin Faisal University, Dammam, SAU; 5 College of Medicine, Majmaah University, Al-Majma'ah, SAU; 6 College of Medicine, King Saud Bin Abdulaziz University for Health Sciences, Riyadh, SAU; 7 College of Medicine, Albaha University, Abha, SAU; 8 General Surgery, Al Kharj Military Industries Corporation Hospital, Al-Kharj, SAU

**Keywords:** case report, neurosurgery, colloid cyst, headache, migraine

## Abstract

Headache is a common cause of emergency department (ED) visits. Migraine is a prevalent neurological disorder that is encountered by emergency physicians in day-to-day practice. However, patients with a known history of migraines should be carefully evaluated when presenting with headaches and serious pathologies of headache should be ruled out. We report the case of a 43-year-old woman, with a known history of classic migraine, who presented to the ED with a severe headache. She described the headache as persistent generalized pain. The headache was worse on awakening and bending. The headache did not improve with the use of oral sumatriptan. She reported that the current episode of headache is more severe than her usual migraine headaches. The patient underwent a cranial CT scan which demonstrated a homogenously hyperdense well-defined round lesion located in the midline at the approximate location of the foramen of Monro with prominent lateral ventricles, conferring the diagnosis of the colloid cyst. The patient underwent a right craniotomy with resection of the cyst using the transcallosal approach. Recognition of this important diagnosis is crucial to prevent serious neurological complications by having timely management.

## Introduction

Headache is one of the most common presentations to the emergency department (ED). It accounts for up to 4% of all emergency visits [1]. The presentation of headache often poses a diagnostic challenge because of the wide spectrum of presenting clinical features with the limited time available for investigation in the ED. Primary headache disorders are the most frequent etiologies for headaches in the ED.

Migraine is a prevalent neurological disorder that is encountered by emergency physicians in day-to-day practice. It is characterized by recurrent attacks of headaches. However, patients with a known history of migraines should be carefully evaluated when presenting with headaches and serious pathologies of headache should be ruled out. We present the case of a middle-aged woman, with a history of migraines, who presented with a severe headache due to a colloid cyst, which is a potentially fatal condition if its management was delayed or missed.

## Case presentation

We present the case of a 43-year-old woman, with a known history of classic migraine for the last 20 years, who presented to the ED with a severe headache. Her pain started four days prior to her presentation and progressively worsened in severity. She described the headache as persistent generalized pain, compared with the pulsatile nature of her previous migraine headaches. The headache was worse on awakening and bending. Unlike her usual episodes of migraine, the headache did not improve with the use of oral sumatriptan. She scored the pain as eight out of 10 in severity and it was awakening the patient from sleep. The headache was associated with nausea and recurrent episodes of vomiting. There was no history of preceding head trauma. The patient did not report any history of photophobia, fever, weakness, or loss of consciousness. The patient visited several outpatient clinics who managed her as having tension headache and offered symptomatic treatment only.

She reported that the current episode of headache was different in character and severe than her usual episodes of migraine headaches. Of note, the patient was using sumatriptan for the last eight years. Her past medical history is not significant for any health condition other than migraine. She has not undergone any surgical operation in the past. Her family history is significant for classic migraines in her mother and sister. She is a non-smoker and does not drink alcohol.

Upon examination, the patient looked in pain and distress. She was drowsy but was fully oriented. Her vital signs on presentation were as follows: pulse rate of 114 bpm, blood pressure of 132/78 mmHg, respiratory rate of 18 bpm, temperature of 36.7℃, and oxygen saturation of 99% on room air. Neurological examination revealed grossly intact cranial nerves, no focal motor or sensory deficits, and normal cerebellar examinations. Funduscopic examination showed normal findings. The cardiorespiratory examination was unremarkable. There was no neck stiffness and the meningeal signs were not present. Her laboratory findings revealed a hemoglobin level of 13.9 g/dL, a white blood cell count of 6,500/µL, and a platelet count of 420,000/µL. Other biochemical investigations, including hepatic and renal profiles, were within the normal range.

In view of the aforementioned clinical features, the patient underwent CT of the brain to rule out any space-occupying lesion. The CT demonstrated a homogenously hyperdense well-defined round lesion located in the midline at the approximate location of the foramen of Monro with prominent lateral ventricles (Figure 1). This finding prompted a further investigation with MRI which redemonstrated the lesion as having an increased T1 and iso T2 signal intensity with the mass (Figure 2). Such findings conferred the diagnosis of a colloid cyst.

**Figure 1:** CT head. Cranial CT scan demonstrating a midline round hyperdense lesion located near the foramen of Monro (arrow) with prominent lateral ventricles.

**Figure 2:** MRI brain. MRI demonstrating the mass lesion near the foramen of Monro with increased T1 signal intensity.

The patient was prepared for an emergency neurosurgical operation for excision of the cyst. She had a right craniotomy with resection of the cyst using the transcallosal approach. The patient tolerated the procedure well without any complications. Histopathological examination of the resected cyst showed a ciliated pseudostratified epithelium lining of the cyst (Figure 3). She had complete resolution of the headache and was discharged on the sixth postoperative day.

**Figure 3:** Histopathology. Histopathological image of the resected cyst demonstrating a ciliated pseudostratified columnar epithelium lining.

## Discussion

We presented the case of a middle-aged woman, with a history of migraines, who presented with progressive headache that was diagnosed as having colloid cyst near the foramen of Monro. The colloid cyst is a rare benign tumor accounting for less than 2% of all primary brain tumors [2]. 

The majority of colloid cysts are asymptomatic and are detected incidentally on imaging. The clinical manifestations of colloid cysts include headache, visual disturbances, vertigo, and even sudden death. Such presentations are related to the obstruction of the flow of the cerebrospinal fluid which precipitates the development of hydrocephalus [3]. In the present case, the headache could have been easily attributed to the history of migraines of the patient [1].

The pathogenesis of colloid cysts remains unclear. It is postulated that the cyst could be a paraphysis remnant, which is an embryonic structure at the diencephalon located between the telencephalon hemispheres. However, this theory does not provide an explanation for the colloid cysts which may be found in the frontal lobe and cerebellum [4].

The diagnosis of colloid cysts can readily be made by CT head or MRI brain. On CT imaging, the cyst appears as a rounded hyperdense lesion near the foramen of Monro [2]. The cyst may exhibit calcification. The differential diagnosis of colloid cysts on imaging is broad, including craniopharyngioma, ependymoma, pituitary tumor, and meningioma [1].

The management approaches for colloid cyst excision include craniotomy using transcallosal or transcortical approaches, endoscopic removal, and stereotactic aspiration. The prognosis is good and the recurrence is very rare [3-4].

## Conclusions

A colloid cyst is a rare benign primary brain tumor. Recognition of this important diagnosis is crucial to prevent serious neurological complications by having timely management. Physicians should have a high index of suspicion for secondary causes of headaches in patients with a migraine so that they do not falsely attribute all the episodes of a headache to migraine.
